This article has been retracted.

# rs10499194 polymorphism in the tumor necrosis factor-α inducible protein 3 (TNFAIP3) gene is associated with type-1 autoimmune hepatitis risk in Chinese Han population

**DOI:** 10.1371/journal.pone.0176471

**Published:** 2017-04-27

**Authors:** Enbin Xu, Hailian Cao, Liming Lin, Honglong Liu

**Affiliations:** Department of Gastroenterology, No.404 Hospital of People’s Liberation Army, Weihai, Shandong, China; Sudbury Regional Hospital, CANADA

## Abstract

Previous studies have found that the polymorphisms of tumor necrosis factor-α induced protein 3 (TNFAIP3) were associated with several autoimmune diseases. However, the role of TNFAIP3 polymorphisms in type-1 autoimmune hepatitis (AIH-1) remained unclear. The present study aimed to clarify the association of TNFAIP3 polymorphisms with AIH-1 risk in a Chinese Han population. The TaqMan SNP genotyping assay was used to determine the distribution of TNFAIP3 polymorphisms in 432 AIH-1 patients and 500 healthy controls. The association of TNFAIP3 polymorphisms and clinical characteristic was further evaluated. Five TNFAIP3 polymorphisms (rs2230926, rs5029939, rs10499194, rs6920220, rs582757) were analyzed in the present study. No significant association could be observed between rs2230926, rs5029939, rs6920220, rs582757 and the susceptibility to AIH-1 in Chinese Han population. Compared with wild-type genotype CC at rs10499194, individuals carrying CT genotype had a significantly increased risk for developing AIH-1 (OR = 2.32, 95%CI 1.44–3.74). Under a dominant model, CT/TT carriers have a 140% increased risk of AIH-1 than CC carriers (OR = 2.40, 95%CI 1.50–3.87). The rs10499194 T allele was also found to be significantly associated with AIH-1 risk (OR = 2.41, 95%CI 1.51–3.82). In addition, higher serum ALT, AST levels and more common cirrhosis were observed in AIH-1 patients with T allele (CT/TT) than those with CC genotype. In conclusion, TNFAIP3 rs10499194 T allele and CT genotype were associated with an increased risk for AIH-1, suggesting rs10499194 polymorphism as a candidate of susceptibility locus to AIH-1.

## Introduction

Autoimmune hepatitis (AIH) is an organ-specific autoimmune disease characterized by a progressive necroinflammatory condition of liver, interface hepatitis, hypergammaglobulinemia and production of autoantibodies[1, 2]. AIH could be categorized into at least two major subtypes based on circulating autoantibodies. Type-1 autoimmune hepatitis (AIH-1) is distinguished by the presence of anti-smooth muscle antibodies (anti-SMA) and/or anti-nuclear antibodies (ANA), which is the major form of AIH in adults[3, 4]. Although the exact etiology remained unclear, the combination of susceptible genetic background and environmental factors was identified to contribute to the development of this disease[5]. The human leukocyte antigens (HLA) DRB1 gene is a well-characterized susceptibility gene and previous studies have identified DRB1*0301, DRB1*0401 associated with the genetic predisposition in Caucasian individuals and DRB1*0405 in Asian individuals[6, 7]. Genetic studies looking outside HLA genes have discovered the polymorphisms of cytotoxic T lymphocyte antigen–4 gene (CTLA-4), tumor necrosis factor–α gene (TNF-α) and Fas as potential non-HLA susceptibility gene to AIH-1[8, 9]. Recently, a genome-wide association study (GWAS) of Japanese AIH patients has identified at least 26 candidate AIH susceptibility or resistance regions other than HLA class II loci, while the GWAS of Dutch AIH patients has yielded 9 independent non-HLA susceptibility loci[10, 11]. Nevertheless, none of the associations described to date could account for all instances of disease. As a complex autoimmune disease, there are undoubtedly other genes involved in the genesis of AIH-1.

The TNF-α–induced protein 3 (*TNFAIP3*) gene is located on chromosome 6q23, which encodes a ubiquitin-modifying enzyme. As a deubiquitination protein, A20 participated in nuclear factor κB (NF-κB) signaling pathway and A20 could inhibit NF-κB function by deubiquitination specific NF-κB signal molecules. Previous study demonstrated defects in A20 expression were associated with the development of several human autoimmune disorders[12]. The establishment of myeloid-specific A20-deficient mice demonstrated that A20 knockout could cause spontaneous development of a severe destructive polyarthritis with several features of rheumatoid arthritis[13]. Loss of A20 in B cells could trigger a progressive inflammatory reaction and cause autoimmune pathology[14]. In addition, the previous study also identified A20-mediated control of dendritic cells activation as a vital checkpoint in the development of systemic autoimmunity[15].

Recently, studies have shown that *TNFAIP3* genetic polymorphisms were associated with susceptibility to multiple human autoimmune and inflammatory diseases including rheumatoid arthritis (RA), systemic lupus erythematous (SLE), polymyositis/dermatomyositis and inflammatory bowel diseases (IBDs)[16–19]. However, until now, there is lack of data about the association between TNFAIP3 polymorphisms and AIH-1 patients risk. Therefore, to determine the effect of TNFAIP3 polymorphisms on AIH-1 risk in Chinese Han population, we performed this case-control study and evaluate the potential associations between five TNFAIP3 polymorphisms (rs2230926, rs5029939, rs10499194, rs6920220, rs582757) with AIH-1.

## Materials and methods

### Participants

432 AIH-1 patients from department of Gastroenterology, No.404 Hospital of People’s Liberation Army (Shandong, China) were consecutively enrolled from June 2010 to February 2016 in this case-control study. All patients fulfilled the 1999 revised diagnostic criteria for AIH-1 recommended by International Autoimmune Hepatitis Group (IAIHG)[20]. Patients were excluded if there was histological evidence of cholangitis or non-alcoholic steatohepatittis, or the presence of hepatitis B virus-surface antigen (HBsAg) and hepatitis C virus related RNA. Patients with other causes, such as alcohol or drug use, were also excluded. In addition, 500 healthy and unrelated controls were matched by gender and age to individual AIH-1 patients during the same period. All controls were healthy volunteers defined as asymptomatic individuals without any diagnosed illness and were normal on detailed physical examination. All participants were Han ethnicity from the same region in Shandong of China. The present study was conducted with the approval of the Ethics Committee of No.404 Hospital of People’s Liberation Army (Shandong, China) and written informed consent was obtained from each individual. All procedures were carried according to the principles of the Declaration of Helsinki.

### Clinical and laboratory data collection

Patient demographic and clinical characteristics were collected from medical records including age, gender, age at diagnosis, markers of HBV and HCV, serum levels of ALT, AST, ALP and total bilirubin. A definite diagnosis of autoimmune hepatitis based on the criteria required a pretreatment score exceeding 15, whereas a probable diagnosis required a score between 10 and 15. ANA, ASMA, liver-kidney microsomal 1 antibody (anti-LKM1) and anti-mitochondrial antibody (AMA) were measured, and a titer of more than 1:40 was considered positive for all autoantibodies. None of all AIH-1 patients was seropositive for anti-LKM1 or AMA. Besides, all AIH-1 patients were tested for antibody to hepatitis virus (A, B, C, E). None of these biomarkers could be observed in any of the patients.

### DNA extraction and genotyping

In the present study, we used TaqMan SNP genotyping assay to determine genotypes for TNFAIP3 polymorphisms. Genomic DNA from AIH-1 patients and healthy subjects were isolated using a Genomic DNA kit (Axygen, CA, USA) based on the manufacturer’s instruction. Genotyping of TNFAIP3 polymorphisms (rs2230926, rs5029939, rs10499194, rs6920220, rs582757) were conducted using custom Taqman SNP genotyping assays (C_7701116_10 for rs2230926, C_29431904_10 for rs5029939, C_1575581_10 for rs10499194, C_29431952_10 for rs6920220, C_8300291_10 for rs582757, ThermoFisher, OK, USA). Genotyping and allele analysis were conducted with TaqMan genotyping master mix (ThermoFisher, OK, USA) and an ABI Prism 7900HT genetic detection system following the manufacturer’s instructions. PCR was performed in a final volume of 25 μL including 12.50 μL master mix, 1.25 μL of assay Mix, 11.25 μL of ddH20. PCR condition was set as follows: 95°C for 15 s, 60°C for 1 min, for 40 cycles. Genotype and allele frequencies were calculated based on allelic discrimination plots using automatic allele analysis. Genotyping of HLA-DRB1 alleles was determined using HLA-DRB1 SSP Morgan kit (Texas BioGene, TX, USA). Genotype reproducibility was assessed in 10% duplicate samples and results were 100% concordant.

#### PBMCs isolation and western blotting

Primary blood mononuclear cells (PBMCs) from 6 AIH-1 patients were obtained using Ficoll density gradient centrifugation(Lymphoprep, Norway). Separated PBMCs were resuspended in RPMI1640 medium supplemented with 10% fetal bovine serum (Gibco, USA), 100 units/mL penicillin, and 100 ug/mL streptomycin (Gibco, USA). PBMCs were incubated in a humidified atmosphere of 5% CO2 at 37^°^C. p-IKB were measured by western blotting after stimulating by lipopolysaccharide (LPS, 10ng/ml) for 1 hour. After LPS stimulation, total proteins was obtained using RIPA buffer containing PMSF and the protein concentration was measured by BCA Protein Assay Kit (Beyotime, China). Approximately 10 ug proteins were separated on SDS-polyacrylamide gel and transferred onto PVDF membranes. After blocking with 5% skimmed milk in TBST buffer for 1h, the membranes were incubated with phospho-IkB antibody (1:1000 dilution, CST, #2859, USA) and β-actin antibody (1:2000 diluation, Abcam, ab8227, USA) at 4 oC overnight. Then, the membranes were washed three times with TBST buffer and incubated with secondary antibody for another 2 h at room temperature. After washing, Chemiluminescence kit (Beyotime, China) was used to obtain the signals.

### Statistical analysis

Continuous data were compared between AIH-1 patients and healthy controls using Student’s *t* test or Mann-Whitney’s U test, while categorical data were compared using Chi-square tests. The association between the TNFAIP3 polymorphisms and AIH-1 risk were estimated by odds ratios (ORs) using the logistic regression model. We set 0.2 as an false-positive report probability (FPRP) threshold and assigned a prior probability of 0.1 to detect an OR of 1.50 (risk effect) for the association with rs10499194. Only the significant result with an FPRP value less than 0.2 was considered a noteworthy finding[21]. The deviation from Hardy-Weinberg equilibrium was assessed by using Chi-square tests. All statistical analyses were performed in SPSS 22.0 (SPSS Inc., Chicago, IL, USA). *p* value less than 0.05 was considered statistically significant.

## Results

The demographic and clinical characteristics of AIH-1 patients were described in **Table 1**. There were no significant differences between AIH-1 patients and healthy controls in terms of age and gender. Age at diagnoses onset ranged from 22 to 65 years (41.3 ± 11.2 years). Among all AIH-1 patients, 310 (71.7%) were positive for ANA (>1:40) and 138 (31.9%) for ASMA and 46 (10.6%) for both. 72 (16.6%) AIH-1 patients had liver cirrhosis at the time of diagnosis. 312 (72.2%) patients were diagnosed with definite AIH, and 120 (27.8%) with probable AIH. 66 AIH-1 patients were accompanied with other immune diseases including 42 thyroid disease, 14 inflammatory bowel disease and 10 rheumatic disease.

**Table 1:** Demographic and clinical characteristics of AIH-1 patients and normal controls.

	AIH-1 patients (N = 432)	Normal Controls (N = 500)
Age (Years)	44.3 ± 13.8	45.1 ± 12.7
Gender (Male/Female)	60/376	56/444
Age at presentation (Years)	41.3 ± 11.2	
Concurrent immune disease	66 (15.3)	
IAIHG Score	16.4 ± 2.7	
>15 (n, %)	312 (72.2)	
10–15 (n, %)	120 (27.8)	
ALT (IU/L)	326 ± 277	32 ± 8.5
AST(IU/L)	299 ± 275	24 ± 7.6
Total Bilirubin (umol/L)	48 ±65	
ANA^+^ (n, %)	310 (71.7)	
SMA^+^ (n, %)	138 (31.9)	
ANA^+^/SMA^+^ (n, %)	46 (10.6)	
LKM1^+^ or AMA^+^ (n, %)	0	
Cirrhosis at presentation (n, %)	72 (16.6)	

IAIHG, International Autoimmune Hepatitis Group, only pretreatment scores were analyzed; ALT, alanine aminotransferase; AST, aspartate aminotransferase; SMA, smooth muscle antibodies; ANA, antinuclear antibodies; LKM1, liver-kidney microsomal 1 antibody; AMA, anti-mitochondrial antibody;

The distribution and statistical analyses of TNFAIP3 polymorphisms in AIH-1 patients and normal controls were summarized in **Table 2**. The analysis did not yield any significant deviation from HWE for these five polymorphisms in control groups (P>0.10 for all). A significant difference could be observed in the distribution of rs10499194 between AIH-1 patients and normal controls. Compared with WT genotype CC at rs10499194, individuals carrying genotype CT and allele T had significantly increased risk for developing AIH-1 (OR = 2.32, 95%CI 1.44–3.74; OR = 2.40, 95%CI 1.50–3.87, respectively). Individuals with T allele at rs10499194 had an almost 141% increased risk of AIH-1 development when compared with C allele (OR = 2.41, 95%CI 1.51–3.82). Howver, there is no statistically significant difference in the frequencies of rs2230926, rs5029939, rs6920220, rs582757 between AIH-1 patient and controls. To determine whether the significant association of rs10499194 polymorphism with disease susceptibility attributed to the overlapping immune disease, we performed the stratification analysis and observed a significant association of rs10499194 polymorphism with susceptibility to AIH-1 patients without other overlapping immune diseases (S1 Table).

**Table 2:** Genotype distribution and allele frequencies for TNFAIP3 gene polymorphisms in both AIH-1 patients and normal controls.

Allele/Genotype	AIH-1 (n, %)	Controls (n, %)	HWE (Controls)	OR (95% CI)	P Value
rs2230926			0.407		
T	826 (95.6)	952 (95.2)		(Reference)	
G	38 (4.4)	48 (4.8)		0.91 (0.59–1.41)	0.74
TT	396 (91.7)	454 (90.8)		(Reference)	
TG	34 (7.8)	44 (8.8)		0.89 (0.56–1.41)	0.63
GG	2 (0.5)	2 (0.4)		1.15 (0.16–8.18)	1.00
TG+GG	36 (8.3)	46 (9.2)		0.90 (0.57–1.42)	0.73
rs582757			0.214		
T	728 (84.3)	832 (83.2)		(Reference)	
C	136 (15.7)	168 (16.8)		0.93 (0.72–1.18)	0.57
TT	312 (72.2)	350 (70.0)		(Reference)	
TC	104 (24.1)	132 (26.4)		0.88 (0.66–1.19)	0.45
CC	16 (3.7)	18 (3.6)		0.99 (0.50–1.99)	1.00
TC+CC	120 (27.8)	150 (30.0)		0.90 (0.68–1.19)	0.47
rs5029939			0.352		
C	818 (94.7)	960 (96.0)		(Reference)	
G	46 (5.3)	40 (4.0)		1.35 (0.87–2.08)	0.19
CC	386 (89.4)	460 (92.0)		(Reference)	
CG	46 (10.6)	40 (8.0)		1.37 (0.88–2.14)	0.17
GG	0 (0)	0 (0)		NS	NA
GG+CG	46 (10.6)	40 (8.0)		1.37 (0.88–2.14)	0.17
rs10499194			0.520		
C	808 (93.5)	972 (97.2)		Reference	
T	56 (6.5)	28 (2.8)		**2.41 (1.51–3.82)**	**0.01**
CC	378 (87.5)	472 (94.4)		Reference	
CT	52 (12.0)	28 (5.6)		**2.32 (1.44–3.74)**	**0.02**
TT	2 (0.5)	0 (0)		NS	NA
CT+TT	54 (12.5)	28 (5.6)		**2.40 (1.50–3.87)**	**0.01**
rs6920220			0.750		
G	726 (84.0)	816 (81.6)		Reference	
A	138 (16.0)	184 (18.4)		0.84 (0.66–1.07)	0.18
GG	306 (70.8)	334 (66.8)		Reference	
GA	114 (26.4)	148 (29.6)		0.84 (0.63–1.12)	0.27
AA	12 (2.8)	18 (3.6)		0.73 (0.35–1.54)	0.46
GA+AA	126 (29.2)	166 (33.2)		0.83 (0.63–1.10)	0.20

To determine the association of HLA-DR alleles and AIH-1 risk, HLA-DR*03:01/*04:05 alleles typing was performed in this cohort of AIH-1 patients. In the analysis of HLA-DR alleles, the frequencies of both HLA-DR*03:01 and *04:05 were significantly increased in AIH-1 when compared with those in controls (p<0.01 for both, **Table 3**). Multivariate logistic regression analysis revealed that T allele at rs10499194 (CT+TT) contributed to the development of AIH-1, independent of HLA-DR*03:01 and *04:05 (OR = 1.78, 95%CI 1.33–2.69).

**Table 3:** Distribution of HLA-DR alleles between AIH-1 patients and normal controls.

HLA-DR alleles	AIH-1 (n = 864 alleles)	Control (n = 1000 alleles)	OR (95%CI)	P Value
HLA-DRB1*03:01	312 (36.1)	237 (23.7)	1.52 (1.26–1.85)	<0.01
HLA-DRB1*04:05	69 (8.0)	52 (5.2)	1.54 (1.06–2.23)	<0.01

Among those patients with rs10499194 T allele, 20 are DRB1*03:01 and 7 are DRB1*04:05.

The association of rs10499194 polymorphism with clinical features of AIH-1 patients were further evaluated. As shown in **Table 4**, the detailed genotype-phenotype analysis showed that patients with CT or TT genotypes had significantly increased serum ALT, AST levels at presentation than those with CC genotype (p<0.01 for both). Besides, there were no significant difference between rs10499194 polymorphism and other clinical features of AIH-1 patients.

**Table 4:** Association of rs10499194 genotypes with clinical characteristics of AIH-1 patients.

	CC (n = 378)	CT+TT (n = 54)	P Value
Age (Years)	44.6 ± 13.7	42.1 ± 14.2	0.21
Gender (Male/Female)	48/330	12/42	0.10
Age at presentation (Years)	41.4± 11.1	40.7± 12.3	0.67
Concurrent immune disease	59	7	0.84
IAIHG Score	16.3 ± 2.7	16.9 ± 3.3	0.14
>15 (n, %)	276	36	0.73
10–15 (n, %)	102	18	0.45
ALT (IU/L)	293 ± 261	561 ± 279	<0.01
AST(IU/L)	271 ± 263	498 ± 273	<0.01
Total Bilirubin (umol/L)	47 ± 64	54 ± 70	0.46
ANA^+^ (n, %)	278	32	0.42
SMA^+^ (n, %)	120	18	0.88
ANA^+^/SMA^+^ (n, %)	39	7	0.64
Cirrhosis at presentation (n, %)	40	32	<0.01

In addition, AIH-1 patients with the CT or TT genotypes at rs10499194 were more likely to have cirrhosis at presentation than those individuals with CC genotype (p<0.01, **Table 4**). 32 of 45 AIH-1 patients with T allele have cirrhosis at entry compared with 40 of 378 those with CC genotype. Multivariate logistic regression analysis also revealed that rs10499194 T allele (CT+TT) was an independent risk factor for liver cirrhosis in patients with AIH-1, independent of age at presentation, gender, ANA/SMA, HLA-DR*03:01 and *04:05 (p<0.05).

Further, we detected p-IkB level in PBMCs after LPS stimulation for 1 hour among AIH-1 patients with TT, CC, TC genotypes. The results were shown in **Fig 1**, p-IkB was increased in AIH-1 patients harboring T allele than C allele, consistent with idea that the patients with the T allele could better activate NF-kB signaling.

**Fig 1:** p-IkB expression in PBMCs from AIH-1 patients after LPS stimulation for 1h. P1/P2: patients (n = 2) with TT genotype; P3: patient (n = 1) with TC genotype; P4/P5/P5: patients with CC genotype (n = 3)

## Discussion

Current evidences suggested that genetic factors have been implicated in the pathogenesis of AIH-1. Although genes located within the HLA region may play a dominant role in the predisposition to AIH-1, HLA alone could not account for the entire genetic predisposition, because about 40% of AIH-1 patients lack those susceptibility alleles[22]. Therefore, previous studies have found susceptibility to AIH-1 may result from genetic variation in immune mechanisms involved in establishing and maintaining self-tolerance, such as CTLA-4, TNF-a, Fas, etc [22, 23]. In the present study, we evaluated the association of five TNFAIP3 polymorphisms with AIH-1 risk and found that rs10499194 T allele and CT genotype were significantly associated with an increased risk for AIH-1. In addition, we observed higher serum ALT, AST levels and more common cirrhosis in AIH-1 patients with rs10499194 T allele.

TNFAIP3 gene encodes the ubiquitin-modifying enzyme A20, a key regulator of NF-kb signaling pathway. Reduced negative regulatory activity of A20 could allow excessive immune activity, causing increased auto-reactivity. Several TNFAIP3 polymorphisms have been identified as risk factors for autoimmune diseases including RA, SLE, primary Sjogren’s syndrome (pSS), etc. In the present study, we chose five polymorphisms mainly based on results previously reported on autoimmune diseases. However, the previous studies yielded controversial results. For example, Zhu did not found significant difference in the frequencies of rs2230926 and rs582757 polymorphisms between RA patients and healthy controls in Chinese population [24]. Conversely, Hao’s study indicated that rs2230926 polymorphism may be a susceptible factor conferring risk for RA in Chinese population[25]. In Korean population, both rs2230926 and rs5029939 were identified to be not significantly associated with RA susceptibility(26). Significantly different frequency of rs5029939 were found in Korean patients with SLE compared with healthy controls[26]. Significant association was also observed for rs2230926 at allelic level in Chinese patients with SLE[27]. However, no significant association between rs2230926, rs5029939 and pSS could be found[28]. In European population, the previous study confirmed that TNFAIP3 rs6920220 polymorphism was associated with RA susceptibility[29]. However, the role of TNFAIP3 polymorphisms in liver disease remain unclear. Zhang’s group have investigated the association of rs2230926 with chronic HBV infection, but did not find significant association between rs2230926 polymorphism with the susceptibility of chronic HBV infection or the progression of HBV-related diseases in Chinese population[30]. Therefore, despite controversial results for those polymorphism across various autoimmune diseases, the true disease-causing variants still remain difficult to pinpoint. Additional association studies in independent cohort are needed to confirm the above findings.

Except for the above four SNPs, we observed a positive association between rs10499194 and AIH-1. rs10499194 is a C to T substitution located in the intergenic region upstream of TNFAIP3. rs10499194 showed highly significant association with AIH-1 in the present study. The genome-wide association scan (GWAS) studies in RA and SLE population gave strong association between rs10499194 polymorphism and these two diseases[31, 32]. Hoffjan’s group got a similar conclusion in multiple sclerosis (MS) population that rs10499194 mutation could contribute to the development of MS[33]. In consistent with our results, Zhang also found a significant association between rs10499194 and RA risk in Chinese Han population[34]. However, there has been some controversy about the association between rs10499194 and other immune-related diseases. For example, previous studies failed to reveal a significant association between rs10499194 and systemic sclerosis in the European Caucasian population[35, 36]. Similarly, no significant association could be observed in patients with allergic rhinitis in Chinese population[36]. In the present study, we found a significant association of rs10499194 mutation and increased risk of AIH-1 development, cirrhosis at presentation. Of course, rs10499194 polymorphism alone could not account for the entire genetic predisposition of AIH-1 due to the lower frequencies of rs10499194 T allele in AIH-1 patients. The combination of several genetic polymorphism contributed to the genetic predisposition of AIH-1 patients such as CTLA-4, TNF-α, etc.

The present study was limited by potential selection bias as a hospital-based case-control study. First, the sample size was relatively small, which may limit accuracy and reliability of results. We used false-positive report probabilities to assess significant findings. As described in S2 Table, we could observe FPRP values of less than 0.2 for the significant associations between rs10499194 polymorphism and AIH-1 risk. However, some stratification analysis still required further validation in larger studies. Second, we could not evaluate the effect of rs10499194 on the prognosis of AIH-1 in its evolution to cirrhosis due to the limit data. We would conduct a multivariable analysis after obtaining the time to cirrhosis of other AIH-1 patients without cirrhosis at presentation in the future. Third, although we observed the association between rs10499194 polymorphism and AIH-1 risk, little is known about its effect on the expression or function of TNFAIP3. The ENCODE project indicates rs10499194 lies within a target site for several transcription factors including JunD, BAF155 (http://genome.ucsc.edu/ENCODE). Thus, functional genetic studies are required to evaluate whether the positive association between rs10499194 and risk for AIH-1 and other autoimmune disease is due to a dysfunction of TNFAIP3 transcriptional regulation. Firth, the accurate time from beginning of AIH-1 to the development of cirrhosis in AIH-1 patients were unclear, so it is impossible to fully exclude the effect of a longer evolution of AIH-1 on the differences in percentage of cirrhosis. Besides, because this work was conducted in a Chinese Han population, the distribution of these polymorphisms in other ethnic groups must be confirmed and data should be replicated in larger independent cohorts of different ethnicities.

In conclusion, the present study revealed that TNFAIP3 rs10499194 T allele and CT genotype were associated with an increased risk for AIH-1, suggesting TNFAIP3 rs10499194 polymorphism as a candidate of susceptibility locus to AIH-1.

## Supporting information

S1 Table The association of rs10499194 polymorphism with susceptibility to AIH-1 without overlapping autoimmune disease; (DOC)

S2 Table False-positive report probability values for association between rs10499194 polymorphism and AIH-1 risk; (DOC)
